# Automated Detection and Segmentation of Exudates for the Screening of Background Retinopathy

This article has been retracted.

**DOI:** 10.1155/2023/4537253

**Published:** 2023-07-14

**Authors:** Jaskirat Kaur, Deepti Mittal, Sharaf Malebary, Soumya Ranjan Nayak, Devendra Kumar, Manoj Kumar, Gagandeep, Simrandeep Singh

**Affiliations:** ^1^Department of Electronics and Communication Engineering, Punjab Engineering College (Deemed to be University), Sector 12, Chandigarh 160012, India; ^2^Electrical and Instrumentation Engineering Department, Thapar Institute of Engineering and Technology, Patiala 147004, India; ^3^Department of Information Technology, Faculty of Computing and Information Technology in Rabigh, King Abdulaziz University, Jeddah 21911, Saudi Arabia; ^4^School of Computer Engineering, KIIT Deemed to be University, Bhubaneswar 751024, Odisha, India; ^5^Department of Computer Science, Wachemo University, Hosaena, Ethiopia; ^6^Faculty of Engineering and Information Sciences, University of Wollongong in Dubai, Dubai Knowledge Park, UAE; ^7^MEU Research Unit, Middle East University, Amman 11831, Jordan; ^8^Computer Science Engineering Department, Chandigarh Engineering College, Mohali, India; ^9^Electronics and Communication Engineering Department, UCRD, Chandigarh University, Mohali, India

## Abstract

Exudate, an asymptomatic yellow deposit on retina, is among the primary characteristics of background diabetic retinopathy. Background diabetic retinopathy is a retinopathy related to high blood sugar levels which slowly affects all the organs of the body. The early detection of exudates aids doctors in screening the patients suffering from background diabetic retinopathy. A computer-aided method proposed in the present work detects and then segments the exudates in the images of retina acquired using a digital fundus camera by (i) gradient method to trace the contour of exudates, (ii) marking the connected candidate pixels to remove false exudates pixels, and (iii) linking the edge pixels for the boundary extraction of exudates. The method is tested on 1307 retinal fundus images with varying characteristics. Six hundred and forty-nine images were acquired from hospital and the remaining 658 from open-source benchmark databases, namely, STARE, DRIVE MESSIDOR, DiaretDB1, and e-Ophtha. The exudates segmentation method proposed in this research work results in the retinal fundus image-based (i) accuracy of 98.04%, (ii) sensitivity of 95.345%, and (iii) specificity of 98.63%. The segmentation results for a number of exudates-based evaluations depict the average (i) accuracy of 95.68%, (ii) sensitivity of 93.44%, and (iii) specificity of 97.22%. The substantial combined performance at image and exudates-based evaluations proves the contribution of the proposed method in mass screening as well as treatment process of background diabetic retinopathy.

## 1. Introduction

Background diabetic retinopathy (BDR), a systemic disease and long-term diabetes complication, is among the leading sources of blindness worldwide [1]. According to International Diabetes Federation, it is estimated that diabetes will affect 438 million people by 2030 [1]. It is a chronic condition that progresses from mild to moderate and then to irreversible form of diabetic retinopathy [2]. Mild form of diabetic retinopathy is characterized by microaneurysms, whereas exudates characterize moderate form of diabetic retinopathy. BDR has no symptoms and usually does not interfere with vision until the diseases progress to serious form of BDR such as proliferative diabetic retinopathy, which is characterized by neovascularization causing irreversible vision impairment or blindness. Furthermore, if BDR is not diagnosed at the initial stages, it may affect other organs of the body and also therapy becomes less successful at this stage of the disease [2]. It is therefore important to diagnose diabetic retinopathy at an early asymptomatic clinical stage.

In accordance with eye specialists, growth in the number and size of exudates is the primary symptom of DR and is used as an indication to identify the stage of DR [3]. Exudates appear as yellowish deposits in retina with sharp and fine edges. They appear in myriad shapes, sizes, and number. The change in shape, size, and number of exudates in a particular image signifies the development of DR. Exudates are mainly characterized as hard exudates and soft exudates as depicted in Figures 1(a) and 1(b), respectively. Hard exudates, associated with moderate BDR, appear as golden orange glassy flakes with defined edges. Soft exudates, on the other hand, are the manifestation of other forms of retinopathy and are light yellow in colour with blurred contours.

The detection of seriousness of DR requires qualitative and quantitative study of changes in exudates. Accurate identification of hard exudates contour is used for the laser photocoagulation process followed for the treatment of BDR. Eye specialists use manual inspection techniques to identify exudates boundaries in retinal fundus images. Manual marking and subsequently segmentation, as well as the precision with which lesions are assessed and associated criteria, are all hugely dependent on the specialist's skill and expertise. As a result, the uncertainty arises from (i) determining the precise borders due to various shapes and intensities, which may contribute to confusion, and (ii) the probability of missing exudates of a few pixels. Furthermore, manually scanning each retinal fundus image becomes tedious resulting in fatigue. Besides that, many patients are unable to receive effective care due to high costs of tests and scarcity of specialists. Thus, accurate identification of hard exudates contours is one of the primary tasks required for the detection of DR and subsequently treating it. Therefore, it is necessary to develop an exudates identification system to aid eye specialists, which will be beneficial in lowering the expense of specialists and eliminating the ambiguity related to manual marking. Moreover, exudates identification is beneficial not only for diagnosis but also for recovery preparation. Therefore, a computer-aided exudates identification and segmentation method of exudates for the diagnosis of BDR has been proposed in this research work. The rest of the article is organized as follows.  Section 2 describes the related work in detail on recent technologies in identification of background diabetic retinopathy.  Section 3 details the retinal datasets used in this work.  Section 4 is about the gradient-based methodology proposed for the segmentation of exudates.  Section 4 describes results and discussion, followed by conclusion in Section 5.

## 2. Related Work

In order to evaluate the diagnostic capacity of the exudates identification and segmentation methods proposed in literature, two types of assessment criteria are used, namely, number of exudates-based assessment and retinal fundus image-based assessments [4].

*Number of exudates-based assessment*: each spot of exudates in retinal fundus image comprises a number of pixels and single infected image may contain one or more than one spots. These spots are segmented by applying exudates identification and segmentation method on retinal fundus images. The assessment of the segmentation results is carried out by comparing results pixel-wise with the reference markings by specialists using mathematically significant performance measures. The assessment results on exudates-based assessment should depict better performance as precise segmentation is necessary for the treatment planning of BDR.

*Retinal fundus image-based assessment*: the major goal of retinal image-based assessment is to identify the occurrence or nonoccurrence of exudates to check any incidence of BDR or not. The results are simply dependent on the occurrence or nonoccurrence of exudates in the fundus. Image-based assessment is mainly carried out by correctly identifying retinal fundus images with exudates and nonexudates. This type of assessment is mainly used for clinical purposes, as the precise number of pixels is not significant from screening standpoint.

The image-based assessment method evaluates the method's ability to distinguish between images with the occurrence or nonoccurrence of exudates. However, if the method does not have the capacity to identify contours of exudates, it demonstrates weak performance. Thus, in order to evaluate the method, it is necessary to evaluate the pixel level segmentation results, but it will provide more precise results than image-based assessment. Therefore, both the assessment criteria are key part in judging in the diagnostic capability of the method as well in clinical systems.

A number of computer-aided methods for the identification and then segmentation of hard exudates have been developed to aid ophthalmologists for the detection of DR [5–22]. The first effort using multilevel thresholding was done by Phillips et al. to detect and segment hard exudates [5]. Ege et al. modified the method designed by Phillips et al. by using combination of various algorithms, namely, thresholding, region growing, and template matching algorithms [6]. This method also applied a classifier to categorize hard exudates from other pathological structures present in retinal fundus image. Another approach was suggested by Sanchez et al. in which mixture model using clustering was applied to segment hard exudates [7]. Analogously, fuzzy C-means based method was developed by Yazid et al. to discriminate pixels based on background, blood vessels, and hard exudates pixels [8]. The major disadvantage of all these methods is that these methods use the criteria that exudates have the highest intensity value as compared to other parts of retinal fundus image and use on intensity-based features to segment exudates. Also, these methods are tested on a limited number of images and thus cannot be generalized to retinal images captured using different cameras or datasets. Thus, such methods do not work well for varying type of images having different intensity values corresponding to exudates.

Various morphology-based methods were proposed in literature to identify and then segment exudates from retinal fundus images. Walter et al. segmented exudates and other structures present in retinal images based on morphological operators [9]. Numerous methods were proposed to detect and then segment exudates by first eliminating retinal blood vasculature and optic disk from the retinal fundus images [9–11] resulting in increase in accuracy. However, these methods were not able to segment landmark structures of retinal images such as optic disk and blood vasculature with different shapes and sizes. In order to overcome these disadvantages, Sopharak et al. designed a clustering and morphological processing-based two-step method for the segmentation of hard exudates [12]. Following this development, Welfer et al. applied morphological operators to improve the variations of colours inside retinal fundus images [11]. This technique was applied based on the fact that exudates are brighter as compared to the other regions of the retinal fundus image. Subsequently, the authors applied thresholding along with subtraction maxima transformation technique to segregate exudates from background. However, exudates were not precisely detected and resulted in low sensitivity and high spurious responses. In order to improve the sensitivity, Zhang et al. discarded all the anatomical and other structures from retinal fundus images apart from exudates [13]. Exudates pixels were detected using random forest classifier followed by mathematical morphological operators. The main benefit of mathematical morphology-based approaches is that they have the ability to remove landmark structures such as optic disk and blood vessels from retinal fundus images. However, these methods will not be generalized due to their incapacity of detecting landmark structures of varying shapes and sizes which in turn result in false responses.

Numerous researchers proposed hybrid methods using varying types of supervised approaches to segment hard exudates effectively [14–17]. Clustering approaches work on the premise of collecting pixels corresponding to exudates. Majority of these approaches are followed by supervised algorithms to segregate correctly and incorrectly detected exudates pixels during clustering process. Combination of clustering and morphology approach for the detection of exudates was initially applied by Sopharak et al. on a very limited database of forty retinal images [12]. The method resulted in improved exudates-based sensitivity but very high processing time per image made it inappropriate for practical usage. In order to further improve the medical significant parameters for exudates detection, Osareh et al. first applied enhancement based on intensity values present in retinal images, then clustering algorithm and finally neural network to precisely segregate exudates from other regions of retinal image [14]. The major development was then brought by Niemeijer et al. wherein all the bright regions of the retinal fundus images were differentiated into hard exudates, soft exudates, and drusen [15]. They employed probability-based method to first determine separate bright regions and subsequently classify them into different bright lesions structures. Similar method to differentiate various bright lesions using feature extraction using sparse coding was developed by Sidibe et al. However, small bright regions were not detected by the proposed method. The main limitation of the abovementioned methods is that they are extremely reliant on the type of exudates structures used for training the algorithms.

Lately, deep learning approaches are being applied on retinal fundus images for the identification and segmentation of lesions present in the retina. The deep learning approaches have an advantage of automatic feature extraction on huge number of images. Recently, numerous methods were developed for the detection of exudates and also they achieved promising results [18–21]. Many researchers used convolutional neural network algorithms for improved accuracy of exudates detection [22–25]. However, they resulted in low sensitivity indicating a smaller number of correctly detected exudates pixels. Lately, a number of deep learning methods are also being developed for disease detection from CT and X-ray images [26, 27]. Last year, convolutional neural network-based methods were used for the detection of leaf diseases and COVID-19 detection [28, 29]. The prime concern while using deep learning network is the requirement of large volumes of data and resources for training. Therefore, in this research work, a robust method is designed for the detection of exudates by (i) identifying the true contours of exudates by applying gradient-based approach, (ii) elimination of suspected false exudates pixels by labelling the connected candidate exudates pixels, and (iii) linking the edge pixels for the boundary extraction of exudates. The main part is that the developed algorithm is evaluated on open source datasets such as STARE and DRIVE [21, 22]. High sensitivity/specificity/accuracy of 95.345/98.63/98.04% in the identification of exudates boundaries contributes to early detection of patients with DR especially in rural areas.

The proposed method includes the following three steps: initially the exudates regions are enhanced using enhancement algorithm and also by eliminating artifacts present in the images captured with fundus cameras; in the next step, candidate exudates pixels are detected by applying gradient and linking based method. Lastly, the proposed method was validated by medically significant performance measures such as sensitivity, specificity, and accuracy. To demonstrate the generalisation capacity of the proposed method and applicability for practical usage, the suggested technique is created and evaluated using retinal images obtained from eye hospital as well as four different open-source benchmark databases, each with individual features such as capture device, area acquired, angle of acquisition, and resolution. The exudates segmentation results attained are then utilized by the eye specialists for the recovery planning of BDR. To summarize, the designed approach is intended to assist eye specialists in finding the severity of the disease and deliver higher accuracy.

## 3. Materials

Retinal fundus images database in the present research work is captured from two platforms: 649 retinal images from eye hospital and 658 retinal images from four open-source benchmark databases. The purpose of using these images from variety of platforms is to test the efficiency of the proposed exudates identification and segmentation method to be independent of different variations in images. Open-source benchmark datasets used are STARE, MESSIDOR, DIARETDB1, and e-Ophtha [30–33]. The detailed overview of all the datasets used in this work along with their reference markings is provided below.

### 3.1. Retinal Images Acquired from Eye Hospital

Between March 2019 and December 2019, 649 retinal images of various intensities, resolutions, contrast, and clarity were obtained from SGHS Hospital, Punjab, India. A total of 375 images comprise hard exudates, 119 with other pathological structures and the remaining with no pathology. These images were taken from Topcon fundus camera, which has the resolution of 3218 × 2138 at an angle of 45°. The reference markings of exudates were provided by the eye specialists. These annotations were used as reference to compute the performance of the proposed method. The clinical supervisor provided the ethical approval to carry out this scientific study.

### 3.2. Open-Source Benchmark Databases

Open-source benchmark datasets have varying aims, attributes, and degree of comprehensiveness as discussed below:

- MESSIDOR dataset: MESSIDOR database comprises of 1200 retinal images acquired using Topcon camera with different resolutions at an angle of 45° [30]. Four hundred images were shortlisted for the present research work comprising of 274 nonpathological images and 126 comprising hard exudates. It provides only the image-based assessment analysis for the detection of DR. Even though it does not provide manual markings, it is a significant source considering the number of accessible images. Thus, to assess the results on these images, manual markings were created by the eye specialists.
- DIARETDB1 dataset: it contains 89 images taken with a fundus camera at an angle of 50° [31]. Eighty-four images out of 89 exhibit minor symptoms of DR, such as exudates, whereas the other 5 are nonpathological retinal images. This dataset was the first dataset comprising reference markings from eye specialists. These markings, on the other hand, solely comprise the enclosures of the pathological regions, and exact markings were generated in the proposed work.
- STARE dataset: a total of 400 images comprise hard exudates and other pathological structures such as red lesions of various shapes and sizes [32]. These images are captured with the Topcon camera which has the resolution of 605 × 700 at an angle of 35°. Image-based DR detection assessment of each retinal image is provided, but does not include reference markings to assess the method based on number of exudates-based assessment. Therefore, in order to assess the exudates-based performance of the proposed method, an eye specialist annotated the contours of the lesions of 96 retinal images having variety of attributes.
- e-Ophtha EX dataset: it contains 82 images comprising 47 pathological and 35 nonpathological images [33]. Retinal images with varying sizes and shapes of exudates and captured at varying resolutions from OPHIDAT medicine centre are present in this database. Furthermore, e-Ophtha database in the sole database providing exudates-based assessment of lesions, which is useful for comparing the efficacy of various exudates identification methods present in literature.

*Reference markings of exudates*: open-source benchmark databases do not comprise exact exudates markings or these annotations are no accurate to compute the performance related to exudates-based assessment. As a result, reference markings of all the images from different datasets are created under the supervision of eye specialists to precisely analyse the performance of the proposed method.

## 4. Methods

The proposed algorithm in this work, as depicted in Figure 2, is comprised of the following stages, such as (i) enhancement of retinal fundus images, (ii) candidate exudates contour detection, and (iii) precise segmentation of exudates.

### 4.1. Enhancement of Retinal Images

To enhance the quality of retinal fundus images for the accurate identification of exudates, it is necessary to remove artifacts in retinal images. These artifacts appear in retinal images due to several aspects such as inappropriate lighting of retinal fundus image, blur, focus, etc. These factors highly contribute to degrading the quality of retinal images. Degraded images can further result in inaccurate detection of retinal diseases. Thus, enhancement of images prior to the identification of exudates is an essential step. The algorithm developed for the enhancement of retinal images comprises three steps: (i) multiplicative transformation for elimination of artifacts due to improper lighting, (ii) channel selection for maximum intensity selection, and (iii) Weierstrass transformation for elimination of blur.

#### 4.1.1. Multiplicative Transformation

Dependency of many factors related to camera, field of view, and expertise of the clinician results in varying types of artifacts in retinal fundus images. These factors result in variation of intensity in varying parts of retinal fundus images. Therefore, in the present work, multiplicative transformation is applied to eliminate the variation of intensity range and enhancing contrast in different parts of retina. In the proposed method, the retinal fundus image *I* (*x*, *y*) is considered as a function of lighting *l* (*x*, *y*) and reflectance components *r* (*x*, *y*) shown in

(1) $$\begin{array}{c} I\left(x,y\right)=1\left(x,y\right).r\left(x,y\right). \end{array}$$

Lighting component of retinal images represents smooth areas corresponding to low frequency and reflectance components represent high frequency components. High frequency components represent the details present in retinal image and thus need to be preserved. Therefore, in order to separate varying frequency components, the Fourier transform (FT) is applied on the image as shown in

(2) $$\begin{array}{c} FT\left[I\left(x,y\right)\right]=FT\left[\ln\left\{1\left(x,y\right)\right\}\right]+FT\left[ln\left\{r\left(x,y\right)\right\}\right]=FTl+FTr, \end{array}$$

where *FT *[ln {*l* (*x*, *y*)}] and *FT* [ln {*r *(*x*, *y*)}] are the *FT* of lighting and reflective components, respectively.

In the next step, the Fourier transform of the retinal image is filtered using maximally flat magnitude filter *M*(*s*, *t*) given in

(3) $$\begin{array}{c} M\left(s,t\right)=1-\frac{1}{1+{\left(s^{2}+t^{2}/a\right)}^{n}}, \end{array}$$

where the denominator of the filter represents the rate of change of frequency range from pass to cut-off range. Further, the transformed image is represented as

(4) $$\begin{array}{c} I\left(s,t\right)=\left\{M\left(s,t\right)FTl\left(s,t\right)\right\}+\left\{M\left(s,t\right)FTr\left(s,t\right)\right\}. \end{array}$$

In the last step, the resultant image is then converted from the frequency domain by applying inverse Fourier transform resulting in preprocessed image. The image is finally termed as *I*_*P*_(*x*, *y*).

#### 4.1.2. Channel for Maximum Intensity

The preprocessed retinal image contains RGB components. Among them, the green component represents the maximum intensity with respect to other structures present in retinal images and is thus selected for further processing.

#### 4.1.3. Weierstrass Transformation

The blur present in retinal fundus images has a distribution similar to Weierstrass transformation [34]. Hence, it is removed by using the smoothing Weierstrass filter. The final enhanced image after the application of Weierstrass filter is thus represented as *I*_*PE*_(*x*, *y*).

### 4.2. Candidate Exudates Contour Detection

Exudates contour identification is the initial and significant tasks in the precise tracing of exudates edges. In order to identify the exudates contour, the following steps are designed in the proposed work.

#### 4.2.1. Gradient Calculation

The enhanced image obtained in the previous step is first passed through the Sobel edge detection filter to calculate the intensity variation using Del operator in both directions of Cartesian coordinates I_PEH_ and I_PEV_, respectively. The edge images obtained for both directions are used to calculate amplitude *I*_*PEamp*_(*x*, *y*) and angle *I*_*PEang*_(*x*, *y*).

(5) $$\begin{array}{c} I_{PE}\left(x,\;y\right)=\left[\begin{array}{c} I_{PEH}\\ I_{PEV} \end{array}\right]=\left[\begin{array}{c} \frac{\partial I_{PE}}{\partial x}\\ \frac{\partial I_{PE}}{\partial y} \end{array}\right],\\ I_{PEamp}\left(x,y\right)=\sqrt{I_{PEH}^{2}\left(x,y\right)+I_{PEV}^{2}\left(x,y\right)},\\ I_{PEang}\left(x,y\right)=\tan^{-1}\frac{I_{PEV}}{I_{PEH}}. \end{array}$$

#### 4.2.2. Preservation of Maximum Intensity Pixels in Neighbourhood

The edge images obtained in both directions are examined to eliminate unnecessary pixels not corresponding to exudates edges. The elimination process is carried out by analysing the entire image to determine whether it belongs to maximum intensity in the neighbourhood or not. It is done by comparing the pixel under consideration with all the other pixels of the neighbourhood. If the intensity value of the pixel under consideration is highest, then the pixel is kept otherwise eliminated.

#### 4.2.3. Elimination of Weak Exudates Pixels by Contour Tracing

The resultant image of the last stage contains candidate exudates pixels. However, the application of the last step may result in false exudates pixels due to variation of intensities and artifacts in retinal images. In order to segregate the false exudate pixels, a dynamic thresholding method is designed in this work. The amplitude image *I*_*PEamp*_(*x*, *y*) is threshold by choosing two set of threshold values, namely, higher and lower threshold values, respectively. If the intensity value of *I*_*PEamp*_(*x*, *y*) is more than the higher threshold value, pixel is preserved and termed as confirmed exudates pixels. On the other hand, if the intensity value of *I*_*PEamp*_(*x*, *y*) is less than the lower threshold value, pixel is termed as false exudate pixel and eliminated. Also, if the pixel intensity value is more than the lower threshold value and less than the higher threshold value, the pixel is termed as weak exudates pixel. The decision on such pixels is taken based on the fact of whether these pixels are connected to confirmed exudates pixels or not. If they are connected, then these will be preserved along with confirmed exudates pixels; otherwise they will be eliminated.

### 4.3. Precise Segmentation of Exudates

The edges obtained in the previous step are comprised of the candidate exudates pixels. The pixels obtained in the previous step are broken or not connected due the nature of filters used. However, in order to extract the precise boundary of exudates, it is significant to link the exudates pixels extracted in the last step. Therefore, the steps followed to extract the exudates are the following.

#### 4.3.1. Exudates Edge Diminishing

The candidate exudates pixels forming the exudates edges determined in the last step appear to be broken parts of exudates contours. The true edge contours are connected pixels forming clusters. However, the pixels which are not in the vicinity of the clusters are not the true exudates pixels and are to be eliminated. These insignificant false pixels are eliminated with the help of morphology diminishing operators.

#### 4.3.2. Retrieval of Exudates Corner Points

The exudates edges in retinal images obtained in the previous step occasionally form the closed connected structures. The precise contour of exudates can be obtained only by connecting the corner points of exudates accurately. Therefore, the corner points estimation is necessary to connect the exudates edges. These corner points are retrieved by traversing the 4 × 4 array in the eight directions, as shown below. The corner point pixel is assumed to be in the centre of this array. The array values denoted by “*s*” determine whether the centre pixel is the corner point or not. If at least one of these values is high, i.e., 1, the centre pixel is considered to be the candidate edge pixel; otherwise it is eliminated.

(6) $$\begin{array}{c} \left[\begin{array}{ccc} s & s & s\\ 0 & 1 & 0\\ 0 & 0 & 0 \end{array}\right]\left[\begin{array}{ccc} 0 & 0 & s\\ 0 & 1 & s\\ 0 & 0 & s \end{array}\right]\left[\begin{array}{ccc} 0 & 0 & 0\\ 0 & 1 & 0\\ s & s & s \end{array}\right]\left[\begin{array}{ccc} s & 0 & 0\\ s & 1 & 0\\ s & 0 & 0 \end{array}\right]. \end{array}$$

#### 4.3.3. Marking of Exudates Corner Points and Contour Detection

The corner points of exudates retrieved in the previous step are marked to connect the exudates pixels accurately. A same mark is allocated to the set of exudates pixels depicting similar characteristics. The breaks in the exudates structures are linked by assessing the spatial properties of the corner points.

Lastly, the contour of exudates is detected by connecting the segments of exudates identified. Exudates segments are connected by neighbourhood analysis method. The designed method comprises 3 steps:

1. Examine the features of exudate pixels in the neighbourhood of each marked exudate pixel.
2. Pixels having the similar features are connected, resulting in forming the contour of exudates.
3. Exudates pixels are connected if the difference between magnitude and angle between pixels under consideration is less than the predetermined magnitude and angle threshold, respectively.

## 5. Results and Discussion

The proposed exudates identification and segmentation method is designed and realized in MATLAB version 2018a on a PC with Intel Core i7 processor. Retinal images from hospital and four open-source benchmark databases, as mentioned earlier, are utilized to enumerate the performance of the proposed computer-aided method. A series of experiments were conducted to adjust the threshold values range at different steps. The optimal intensity thresholds are the ones that achieve best sensitivity/specificity combination. Increase in sensitivity indicates the correct detection of bright as well as subtle exudates, whereas higher specificity shows that the method does not recognize a nonexudates pixel as an exudates pixel. A total of 1307 retinal images comprising 525 nonpathological, 623 with exudates, and 157 with other retinopathies with different characteristics such as colour, location, resolution, etc. are used in this work. The performance validation of the designed method is done by (i) visual evaluation of expert ophthalmologist and (ii) medically important statistical measures such as sensitivity, specificity, accuracy, and positive predictive value [35]. These statistical measures are enumerated at two different levels, i.e., image-based assessment and exudates-based assessment. Image-based assessment differentiates images based on the existence or nonexistence of exudates and thus aids in mass screening of patients with background diabetic retinopathy. However, exudates-based evaluation discriminates exudates pixels from nonexudates pixels. This evaluation is primarily used in treatment process of diabetic retinopathy wherein precise boundary exudate markings are required for laser photocoagulation.

### 5.1. Visual Evaluation of Expert Ophthalmologist

Figures 3(a)–3(c) are arbitrarily selected images to depict the performance of the designed method. Figures 3(a) and 3(b) depict the presence of exudates in images of retina. Exudates in these retinal fundus images have clear boundaries and clearly separate themselves from the background. The exudates segmentation results by the proposed computer-aided method, in Figures 3(d) and 3(e), are very alike to the ground truths provided by the experts. Careful analysis of Figures 3(d) and 3(e) shows that the designed method segments minute exudates which were not even marked by experts.  Figure 3(c) shows the exudates with the fuzzy boundaries. The segmentation results by the proposed method in Figure 3(f) depict that few exudates pixels are missed, whereas few are wrongly detected. This is due to the fact that, in these images, exudates pixels mix with the background resulting in fuzzy boundaries. Also, the ophthalmologists opined that out of 623 retinal fundus images 612 images are segmented in such a way that it can be used for screening as well as treatment process. Out of the remaining 11 retinal fundus images, 9 were with fuzzy exudates boundaries and can only be used for mass screening and the segmentation results of 2 images were not suitable and hence rejected.

### 5.2. Performance Evaluation by Medically Important Statistical Measures

Performance evaluation of the proposed computer-aided method in terms of medically significant performance parameters at two levels, i.e., exudates-based and image-based, on 1307 retinal fundus images is tabulated in Table 1.

#### 5.2.1. Number of Exudates-Based Assessment

In this evaluation, medically significant statistical measures are computed by comparing the ground truths of exudates boundary pointed by the expert ophthalmologist with the exudates segmentation results at exudates-based level by the proposed method. Table 1 clearly demonstrates that the designed method attains the average sensitivity, specificity, and accuracy of 91.21%, 96.21%, and 94.12% on the STARE dataset, respectively. The exudates segmentation outcomes of the STARE dataset are in near proximity to the exudates segmentation results of Kaur and Mittal [35]. Additionally, the overall segmentation results of the designed computer-aided method indicate clearly the substantial performance of the proposed exudates segmentation method. The bar graphs in Figure 4 depict the mean sensitivity, specificity, and accuracy along with the deviations around the mean value. These bar graphs depict the overall high value of particularly sensitivity of 93.44% and the mean deviation of 2.63% as compared to the method of Kaur and Mittal which showed the sensitivity of 88.85% and deviation of 4.73%. On comparing other parameters in Figure 4, it can be examined that the designed method has the substantial contribution in attaining the overall mean specificity and accuracy of 97.22% and 95.68%, respectively. Also, the mean deviation values are also comparable to the method proposed by Kaur and Mittal [35]. From Table 1, the proposed computer-aided method clearly outperformed all the exudates-based segmentation methods, thus rationalizing the segmentation results.

#### 5.2.2. Retinal Fundus Image-Based Assessment

In this evaluation, medically significant statistical measures are computed by comparing the number of images marked by expert ophthalmologist as pathological, i.e., images with the incidence of exudates, and normal images with those of the designed method results. The overall mean sensitivity, specificity, and accuracy of 95.345%, 98.63%, and 98.04%, respectively, for image-based validation demonstrate the ability of the designed computer-aided method to discriminate images based on the occurrence and nonoccurrence of the exudates in contrast to the methods reported in literature. However, the method proposed by [41] shows 100% image-based evaluation results for all statistical measures. The main limitation of [41] is that the method has been validated on only 45 retinal fundus images. Table 1 depicts that the overall sensitivity, specificity, and accuracy on the retinal images acquired from hospital are 97.45%, 99.76%, and 98.65%, respectively, for the image-based assessment criteria. These results clearly indicate the capability of the proposed method to discriminate retinal images based on the absence or presence of exudates. Moreover, it can also be observed that the proposed method shows the best performance for sensitivity, specificity, and accuracy for clinical images acquired. Conclusively, the proposed method has achieved high values of medically significant statistical measures in comparison to the other methods. Therefore, subjectively as well as objectively, the designed exudates segmentation method is robust in contrast to the exudates segmentation methods proposed in literature.

## 6. Conclusion

A new exudates segmentation computer-aided method for the detection of background diabetic retinopathy has been designed in the present research work. The designed computer-aided method efficiently segments exudates in images of retina as it involves the steps such as (i) enhancement of retinal fundus images, (ii) candidate exudates contour detection, and (iii) precise segmentation of exudates. The performance of the designed exudates segmentation computer-aided method has been validated on 1307 images of retina from two sources, namely, eye hospital and four open-source benchmark databases. Results of the visual evaluation of the expert ophthalmologist are supported by the results obtained by the medically significant performance parameters, namely, exudates-based evaluation and image-based evaluation. The exudates-based evaluation outcomes specify the high precision of the designed method in correct detection of exudates pixels with sensitivity of 93.44%. The exudates-based evaluation results thus reveal the capability of the designed method in treatment process of background diabetic retinopathy. The specificity of 97.22% shows the ability of the method in successfully differentiating the exudates pixels from the nonexudates pixels. In addition, the proposed method outperformed another recent exudates segmentation method in terms of image-based evaluation with the accuracy of 98.04%. Therefore, the proposed method shows its potential in mass screening of patients with background diabetic retinopathy. Lastly, it can be highlighted the proposed computer-aided method may be used to assist the expert ophthalmologists in the preliminary detection and diagnosis of background diabetic retinopathy.

## Figures and Tables

**Figure 1:** Retinal images showing (a) hard exudates and (b) soft exudates.

**Figure 2:** Layout of the proposed exudates segmentation method.

**Figure 3:** Original retinal images and their corresponding segmentation results by the proposed exudates segmentation method. (a–c) Original retinal fundus images from online datasets. (d–f) Results of proposed exudates extraction methods. (g–i) Reference ground truths.

**Figure 4:** Summary of medically important statistical measures for (a) the proposed exudates segmentation method and (b) the method proposed by Kaur and Mittal on open-source datasets.

**Table 1:** Performance evaluation of the proposed method at exudates-based and image-based levels.

Author	Datasets	Number of retinal fundus images used	Exudates-based assessment (%)			Image-based assessment (%)		
			Sensitivity	Specificity	Accuracy	Sensitivity	Specificity	Accuracy
Reza et al. [36]	STARE DRIVE	20	94.3%	100%	----	----	----	----
Yazid et al. [8]	STARE	15	97.8%	99%	----	----	----	----
Jaya et al. [37]	Clinical	200	94.1%	90%	93%	----	----	----
Welfer et al. [11]	DIARETDB1	89	70.4%	98.84%	----	----	----	----
Niemeijer et al. [15]	Clinical	300	----	----	----	95%	86%	----
Youssef et al. [38]	Clinical	7	----	----	----	80%	100%	----
Lahmiri et al. [39]	STARE	45	----	----	----	100%	100%	100%
Osareh et al. [14]	Clinical	142	93%	94.1%	----	95%	88.9%	----
Gracia et al. [40]	Clinical	117	88.08%	----	----	100%	83.95%	93.53%
Sanchez et al. [7]	Clinical	80	90.2%	----	----	100%	90%	----
Harangi et al. [41]	DIARETDB1	89	63%	85%	----	89%	----	----
Kaur and Mittal [35]	Multiple datasets	1307	88.85%	96.15%	93.46%	94.62%	98.64%	96.74%
Khojasteh et al. [42]	DIARETDB e-Ophtha	284	----	----	----	96%	98%	98%
Kusakunniran et al. [43]	DIARETDB1 e-Ophtha EX	284	56.4%	99.9%	99.8%	----	----	----
Balasubramanian et al. [44]	RIM-ONE	15	----	----	----	----	----	97.8%
Proposed method	**Clinical**	**649**	**95.67%**	**98.23%**	**97.24%**	**97.45%**	**99.76%**	**98.65%**
	**MESSIDOR**	**400**	**91.21%**	**96.21%**	**94.12%**	**93.24%**	**97.49%**	**97.43%**
	**e-Ophtha EX**	**72**	**93.47%**	**94.57%**	**93.47%**	**93.87%**	**94.28%**	**93.82%**
	**DiaretDB1**	**70**	**92.47%**	**98.84%**	**96.78%**	**96.78%**	**97.28%**	**99.02%**
	**STARE**	**86**	**95.38%**	**96.98%**	**96.12%**	**94.98%**	**93.28%**	**97.98%**
	**DRIVE**	**30**	**98.89%**	**97.23%**	**98.23%**	**95.23%**	**95.23%**	**97.32%**
	**OVERALL**	**1307**	**93.44%**	**97.22%**	**95.68%**	**95.345%**	**98.63%**	**98.04%**

## Data Availability

Data are available on request to the first author (Jaskirat Kaur).

## Abbreviations

BDR: Background diabetic retinopathy
DR: Diabetic retinopathy
*FT*: Fourier transform
*FT* [ln {*l* (*x*, *y*)}]: Fourier transform of lighting component
*FT* [ln {*r* (*x*, *y*)}]: Fourier transform of reflective component
*I* (*x*, *y*): Retinal fundus image
*I*_*P*_(*x*, *y*): Preprocessed image
*I*_*PE*_: (*x*, *y*). Enhanced image after the application of Weierstrass filter
*I*_*PEH*_: Edge image obtained after application of Del operator in horizontal direction
*I*_*PEV*_: Edge image obtained after application of Del operator in vertical direction
*I*_*PEamp*_: (*x*, *y*) Amplitude of the of the edge image obtained
*I*_*PEang*_: (*x*, *y*) Angle of the of the Edge image obtained
*l* (*x*, *y*): Lighting component
*M* (*s*, *t*): Magnitude filter
*r* (*x*, *y*): Reflectance component.
